The article "Influence of a novel histone deacetylase inhibitor panobinostat (LBH589) on the growth of ovarian cancer" was published in 2016. Journal: J Ovarian Res.

# Influence of a novel histone deacetylase inhibitor panobinostat (LBH589) on the growth of ovarian cancer

**DOI:** 10.1186/s13048-016-0267-2

**Published:** 2016-09-15

**Authors:** Leslie A. Garrett, Whitfield B. Growdon, Bo R. Rueda, Rosemary Foster

**Affiliations:** 1 Division of Gynecologic Oncology, Department of OB/GYN, Beth Israel Deaconess Medical Center, 330 Brookline Ave, Kirstein 3rd Floor, Boston, MA 02215 USA; 2 Division of Gynecologic Oncology, Department of OB/GYN, Massachusetts General Hospital, 55 Fruit Street, Yawkey 9, Boston, MA 02114-2696 USA; 3 Vincent Center for Reproductive Biology, Department of OB/GYN, Massachusetts General Hospital, 55 Fruit Street, Their 9, Boston, 02114-2696 USA; 4 Harvard Medical School, Boston, MA 02114 USA

**Keywords:** Ovarian cancer, Histone deacetylase inhibitor, Patient derived xenograft model, Conventional chemotherapy

## Abstract

**Background:**

Pre-clinical studies have demonstrated that natural and synthetic histone deacetylase (HDAC) inhibitors can impede the in vitro and in vivo growth of cell lines from a variety of gynecologic and other malignancies. We investigated the anti-tumor activity of panobinostat (LBH589) both in vitro and in vivo as either a single agent or in combination with conventional cytotoxic chemotherapy using patient-derived xenograft (PDX) models of primary serous ovarian tumors.

**Methods:**

The ovarian cancer cell lines OVCAR8, SKOV3 and their paclitaxel-resistant derivatives OVCAR8-TR and SKOV3-TR were treated with increasing doses of LBH589. The effect of LBH589 on cell viability was assessed using the 3-(4,5-dimethylthiazol-2-yl)-2,5-diphenyltetrazolium bromide (MTT) assay. Serially transplanted primary human high-grade serous ovarian adenocarcinoma tissue was utilized to generate xenografts in 6-week old female NOD/SCID mice. The mice were then randomized into one of 4 treatment groups: (1) vehicle control; (2) paclitaxel and carboplatin (P/C); (3) LBH589; or (4) P/C + LBH589. Mice were treated for 21 days and tumor volumes and mouse weights were obtained every 3 days. These experiments were performed in triplicate with three different patient derived tumors. Wilcoxan rank-sum testing was utilized to assess tumor volume differences.

**Results:**

In vitro treatment with LBH589 significantly reduced the viability of both taxol-sensitive and taxol-resistant ovarian cancer cell lines (*p* < 0.01). In vivo treatment with LBH589 alone appeared tumorstatic and reduced tumor growth when compared to vehicle treatment (*p* < 0.007) after 21 days. This single agent activity was confirmed in two additional experiments with other PDX tumors (*p* < 0.03, *p* < 0.05). A potential additive effect of LBH589 and P/C, manifested as enhanced tumor regression with the addition of LBH589 compared to vehicle (*p* < 0.02), in one of the three analyzed serous PDX models.

The article "Influence of a novel histone deacetylase inhibitor panobinostat (LBH589) on the growth of ovarian cancer" was published in 2016. Journal: J Ovarian Res.

**Conclusions:**

Our findings suggest that pan-HDAC inhibition with panobinostat precludes the growth of ovarian cancer cell lines in vitro and PDXs in vivo. Added benefit of LBH589 to standard P/C therapy was observed in one of three PDX models suggesting improved response in a subset of serous ovarian cancers.

## Background

Epithelial ovarian cancer is the second most common, but most lethal gynecologic malignancy in the United States (US) and is estimated to affect approximately 22,280 women and lead to 14,240 deaths in 2016 [1]. Approximately 75 % of patients present with advanced stage disease, a factor largely attributed to the absence of effective screening strategies [2]. At the time of diagnosis, most women will undergo aggressive cytoreductive surgery with the subsequent delivery of platinum based chemotherapy [3]. The combination of carboplatin and paclitaxel is standard first line chemotherapy in the US and, while effective at generating responses in approximately 80 % of women, it is seldom curative [4]. Despite advances in therapy and delivery, recurrence and chemotherapy resistance are still formidable problems as the majority of patients with ovarian cancer who achieve a complete remission with first line platinum-based chemotherapy will ultimately develop recurrent disease that is less responsive to cytotoxic chemotherapy [5]. Finding new molecular targets and exploiting cellular pathways involved in the onset and progression of platinum resistant ovarian cancer will be essential to innovating the treatment of women with this lethal disease [6].

Epigenetic alterations have emerged as key factors in tumorigenesis and may have relevance in the therapy of women with ovarian cancer [7]. Specifically, interfering with gene transcription mechanisms through histone modification may lead to aberrant genetic changes responsible for the development of cancer [8, 9]. During mitosis, histones are modified through acetylation and deacetylation which serve to regulate chromosomal segregation and DNA access to transcription factors [10]. Acetylation causes a conformational change in the histone N-terminal tail resulting in displacement of the histone away from the DNA strand and increased transcriptional activation [11]. Histone deacetylases (HDAC) reverse this process and prevent interactions between transcription factors and DNA [12]. Multiple classes of HDACs have been described and have been shown to exert their effects in various tissues and cellular components [10].

The article "Influence of a novel histone deacetylase inhibitor panobinostat (LBH589) on the growth of ovarian cancer" was published in 2016. Journal: J Ovarian Res.

Recognized as potent epigenetic inhibitors, HDAC inhibitors appear to exert anti-tumor effects through hyperacetylation of histones and demethylation of genomic DNA resulting in reactivation of genes that inhibit proliferation [10, 13, 14]. Both transcriptional and non-transcriptional mechanisms of action have been investigated [15]. Pre-clinical studies using cell lines from a variety of gynecologic [16–18] and other malignancies [19, 20] have demonstrated that natural and synthetic HDAC inhibitors can inhibit tumor cell growth in vitro and in vivo through cell cycle arrest as well as the induction of mitotic defects through histone mediated and histone independent interactions [15]. Investigations utilizing in vitro and in vivo models of ovarian cancer have demonstrated that HDAC inhibition synergizes with conventional chemotherapies to induce potent cytotoxic effects supporting the potential use of this combination in the clinic [18, 21–25]. Early clinical investigations determined that HDAC inhibitors were well tolerated therapeutics with single agent bioactivity against a variety of hematologic malignancies leading to the United States Food and Drug Administration approval of SAHA (Vorinistat) for the treatment of cutaneous T-cell lymphoma [26]. Although only modest single agent activity has been noted in solid tumors in Phase I and II human trials [7, 24, 27–31], mounting preclinical data suggest HDAC inhibition could be effective for patients with ovarian cancer [17, 32]. Relevant in vitro and in vivo models will be required to gain more insight into both the mechanisms of drug action and optimal combinations with conventional chemotherapy [22].

Investigators have observed that HDAC inhibition may be mediated in some cells by modulating expression of the Aurora A serine/threonine kinase [15, 33]. Aurora A is a key regulator of mitotic spindle cell formation and chromosomal segregation and is therefore critical to proper cell cycle progression [34, 35]. Located on chromosome 20q13.2, the *AURKA* gene has been noted to be amplified in several human epithelial tumors and has been an attractive target for developmental therapeutics [36–39]. In ovarian cancer, *AURKA* is amplified in several cell lines and amplification has been shown to correlate with poor prognosis [40, 41]. Additionally, investigators have shown that elevated Aurora A protein expression overrides the checkpoint mechanism that monitors mitotic spindle assembly and is involved in the development of resistance to paclitaxel [42]. Treatment of cancer cells with HDAC inhibitors resulted in a down regulation of Aurora A protein levels suggesting that the most robust responses to HDAC inhibition may be observed in those patients whose tumors exhibit heightened Aurora A expression [15]. Preliminary in vitro data suggests that HDAC inhibition potentiates the effects of Aurora A expression and can sensitize to Aurora kinase inhibitors in ovarian cancer cell line models [43].

The article "Influence of a novel histone deacetylase inhibitor panobinostat (LBH589) on the growth of ovarian cancer" was published in 2016. Journal: J Ovarian Res.

In preliminary studies using the HDAC inhibitors trichostatin A (TSA) and SAHA, we demonstrated significant anti-tumor activity in PDX models of high grade serous ovarian cancer. We sought to explore the possibility that LBH589, a potent inhibitor of class I, II, and IV HDAC enzymes in clinical trial, may act to inhibit tumor cell growth through the degradation of Aurora A. Furthermore, we hypothesized that the administration of LBH589 in concert with conventional cytotoxic chemotherapy would manifest synergistic activity in a subset of serous ovarian cancer PDX models. This investigation sought to provide rationale for pursuing HDAC inhibition in a subset of women with serous ovarian cancer.

## Methods

### Cell culture and cell growth inhibition assay

The human ovarian cancer cell lines OVCAR-8, SKOV3, OVCAR8-TR and SKOV3-TR [44] were grown and maintained in Dulbecco’s Modified Eagle’s Medium (DMEM 1X, 10 % fetal bovine serum [FBS], 1 % P/S). Cells were seeded in triplicate on 24-well plates and then treated with escalating doses of SAHA or LBH589 for 48 h at 37 °C. Cell viability was then assessed by MTT assay as previously described [45].

### Tumor collection and propagation in vivo

Excess human serous ovarian tumor samples were obtained through an IRB approved centralized banking infrastructure at the Massachusetts General Hospital (MGH). Written informed consent was received from all participants. Tumor was enzymatically processed to achieve a single cell suspension and then depleted of hematologic components as described [46]. A specified number of cells were suspended in PBS:Matrigel® (1:1) and injected subcutaneously (s.c.) into 6–8 week old female NOD/SCID mice (Jackson Laboratory, Bar Harbor, ME). Animals were monitored continually to assess tumor formation and size, and euthanized when they became moribund or had excessive tumor burden. All animal experiments were approved by the Massachusetts General Hospital Institutional Animal Care and Use Committee. For continued propagation in mice, the xenograft tumors were excised and enzymatically processed to a single cell suspension. The suspension was depleted of mouse H2K^d+^ cells and the remaining tumor-derived cells were re-injected subcutaneously into new recipient NOD/SCID mice as described [46]. All of the primary human papillary serous ovarian tumors utilized in this study had undergone 4–5 passages in vivo and the serous histology of each was maintained over the serial transplantation process. Animals were housed and maintained in accordance with institutional guidelines.

The article "Influence of a novel histone deacetylase inhibitor panobinostat (LBH589) on the growth of ovarian cancer" was published in 2016. Journal: J Ovarian Res.

### Treatment with LBH589 alone and in combination

Mice bearing matched sized tumors (300–600 mm^3^) from three independent human papillary serous ovarian cancers (OV1, OV2, and OV3) were randomized into four cohorts of six mice each. The four groups were assigned to the following treatment regimens: (1) intraperitoneal (IP) injection of paclitaxel and carboplatin (P/C) vehicle one time per week + IP injection of LBH589 vehicle five times per week; 2) IP injection of paclitaxel (15 mg/kg) and carboplatin (50 mg/kg) one time per week + IP injection of LBH589 vehicle five times per week; (3) IP injection of P/C vehicle one time per week + IP injection of LBH589 (2.5 mg/kg) five times per week; or (4) IP injection of P/C one time per week + IP injection ofLBH589 five times per week. Mice were treated for 21 days with tumor volumes and mouse weights obtained every 3 days. At the end of the treatment period, animals were euthanized and portions of harvested tumors were snap frozen for protein analysis and embedded in paraffin for histological analysis.

### Immunoblotting

For the in vitro cell line experiments, plated OVCAR8 and SKOV3 cells were treated with LBH586 (7.5 nM) or SAHA (2 μM) for 16 h and total cell lysates were prepared. A total of 10–20 μg of protein from each sample was electrophoresed on a precast Tris–Hepes–SDS polyacrylamide gel (Pierce, Thermo Scientific) and transferred onto a PVDF membrane. The membrane was blocked in 5 % non-fat dry milk prepared in TBST. Primary monoclonal antibodies directed against Aurora A kinase, acetylated tubulin and acetylated histone H3 were obtained from Cell Signaling Technology and used according to the manufacturer’s recommendations. Following incubation overnight at 4 °C, each blot was washed, incubated with the appropriate secondary antibody and developed using enhanced chemiluminescence.

### Statistical analysis

Non-parametric Wilcoxan rank sum tests for unpaired samples were used to compare tumor sizes in the LBH589 treatment xenograft experiments. Two-way ANOVA analysis and Student’s t-tests were used to determine the statistical significance of results obtained in the MTT analyses of cell viability. Significance was set at *p* ≤ 0.05. STATA (College Station, TX) v10 software was used.

## Results

### LBH589 reduces ovarian cancer cell viability in vitro

Exposure to increasing doses of LBH589 decreased cell viability of both chemosensitive and chemoresistant ovarian cancer cell lines [44] (Fig. 1, *p* < 0.01). Treatment with 7.5 nM LBH589 led to a 50 % reduction in the viability of OVCAR8 cells while OVCAR8-TR cells were significantly less sensitive to LBH589 (50 % reduction around 7.5 nM, *p* < 0.01). A 50 % reduction in the viability of SKOV3 and SKOV3-TR cells was observed at LBH589 concentrations of 25 nM and 100 nM, respectively (*p* < 0.01). We compared the potency of LBH589 to the only established FDA approved HDAC inhibitor suberoylanilide hydroxamic acid (SAHA, Vorinistat) and observed that the concentrations required for inhibition of OVCAR8 and SKOV3 cell growth were approximately 2-fold less for LBH589. These results are summarized in Fig. 1.

The article "Influence of a novel histone deacetylase inhibitor panobinostat (LBH589) on the growth of ovarian cancer" was published in 2016. Journal: J Ovarian Res.

**Fig. 1:** HDAC inhibition reduces the viability of ovarian cancer cell lines in vitro. The ovarian cancer cell lines OVCAR8 (**a**), SKOV3 (**b**) and their paclitaxel resistant derivatives OVCAR8-TR (**a**) and SKOV-3-TR (**b**) were treated in triplicate with the indicated concentrations of SAHA or LBH589 for 48 h. Relative viability was assessed by MTT assay. Data plotted are mean +/− SEM

### Treatment with LBH589 and SAHA alters acetylated tubulin and Aurora A protein expression in vitro

Acetylated tubulin and acetylated histone H3 are known HDAC targets [47, 48]. We therefore analyzed the effect of LBH589 on acetylation of these proteins to validate that LBH behaves like other HDAC inhibitors and compared any observed effect to that obtained with SAHA. As shown in Fig. 2, treatment with both LBH586 and SAHA led to increased levels of acetylated tubulin and histone H3. We similarly analyzed Aurora A kinase levels following HDAC inhibition. Although Aurora-A kinase was detected in the OVCAR8 cell line, no significant change in its levels was observed following treatment with LBH589. In contrast, SAHA treatment led to a marked reduction in Aurora A kinase levels in OVCAR8. We detected no Aurora A kinase expression in SKOV3 cells.

**Fig. 2:** Effect of in vitro HDAC inhibition on acetylated histone and tubulin. OVCAR8 and SKOV3 cells were treated with 2 μM SAHA, 7.5 nM LBH589 or vehicle for 16 h. Total cellular protein was isolated and subjected to Western blot analysis to determine the relative levels of acetylated tubulin, acetylated histone H3 and Aurora-A kinase. β-actin was used as a protein loading control

### HDAC inhibition blocks the growth of primary human serous ovarian tumor xenografts in vivo

We assessed the single agent activity of LBH589 as well as the potential therapeutic synergy of LBH589 and paclitaxel and carboplatin (P/C) combination therapy. These analyses were carried out with xenografts derived from three individual patient tumors. All of the patients were diagnosed with advanced stage, high grade serous ovarian cancer and had undergone primary upfront surgical cytoreduction (Table 1). To assess the single agent activity of LBH589, we treated mice harboring human serous ovarian cancer xenografts with either LBH589 or vehicle and regularly assessed the effect on tumor volume. Treatment with LBH589 alone appeared tumorstatic when compared to vehicle (OV1, *p* < 0.007; OV2, *p* < 0.03; OV3, *p* < 0.05) after 21 days (Fig. 3).

The article "Influence of a novel histone deacetylase inhibitor panobinostat (LBH589) on the growth of ovarian cancer" was published in 2016. Journal: J Ovarian Res.

**Table 1:** The clinical characteristics of the patients from whom the high grade serous ovarian carcinoma samples were obtained

Patient	Age at diagnosis (Years)	Stage	Grade	Progression free survival (Months)	Overall survival (Months)	Current status
OV1	59	IV	3	22.8	74.4	Deceased
OV2	64.5	IIIC	3	N/A	N/A	N/A
OV3	38.3	IV	3	34.1	86.4	Alive

All patients underwent primary debulking surgery for advanced stage ovarian cancer and had optimal cytoreduction. One patient was lost to follow up and therefore recurrence and overall survival data are not available

**Fig. 3:** Pre-clinical analyses of LBH589 activity in vivo. Separate experiments utilizing PDXs derived from three individual patients are shown. Each evaluated the activity of LBH589 as a single agent and in combination with carboplatin and paclitaxel (P/C) chemotherapy. In all experiments, LBH589 induced statistically significant tumorstasis (*p* < 0.007, *p* < 0.03, *p* < 0.05). In one experiment (OV3), increased tumor regression was observed when LBH589 and P/C were combined (*p* < 0.02)

We then assessed whether LBH589 would have additional antitumor effects when combined with the standard of care chemotherapy regimen of paclitaxel and carboplatin (P/C). The OV3 PDXs demonstrated further tumor regression with the addition of LBH589 to P/C compared to P/C or LBH586 alone, (*p* < 0.02). This effect, however, was not confirmed with the OV1 and OV2 serous PDXs. In the two experiments where LBH589 did not show any additional benefit, treatment with P/C either alone or in combination with LBH589 resulted in complete tumor regression in all animals by day 21. In the majority of treatment arms, the animals lost an average of 10 % of their starting body weight with non-statistically significant weight loss in any arm receiving single agent P/C (*p* < 0.07) or LBH (*p* = 0.06). The most significant weight loss was observed in those animals receiving combination therapy (*p* < 0.005) (data not shown).

## Discussion

These data suggest that single agent HDAC inhibition with LBH589 leads to tumorstatic effects in primary human xenografts derived from patients diagnosed with high-grade serous ovarian cancer. This pattern of tumor inhibition was demonstrated in triplicate across three separate high grade serous tumors obtained from patients who underwent optimal upfront surgical cytoreduction. Combination of LBH589 with conventional cytotoxic P/C, the current platform for the treatment of women with epithelial serous ovarian cancer, resulted in significant tumor regression in one of the analyzed PDX models. These data suggest that that HDAC inhibition may potentiate the activity of cytotoxic therapy in a subset of high grade serous ovarian tumors. These in vivo observations were confirmed by in vitro experiments with immortalized ovarian cancer cell lines OVCAR8 and SKOV3, as well as paclitaxel resistant derivatives of these lines [44] and echoes many recent reports that suggest HDAC inhibition can potentiate conventional and targeted therapeutics.

The article "Influence of a novel histone deacetylase inhibitor panobinostat (LBH589) on the growth of ovarian cancer" was published in 2016. Journal: J Ovarian Res.

Numerous reports have implicated heightened HDAC activity, histone hypo-acetylation and subsequent silencing of tumor suppressor transcription with malignant transformation [49, 50]. Researchers have also proposed that in addition to histone mediated alterations, HDACs may induce DNA independent oncogenic changes to other proteins involved in cell cycle and apoptosis, such as p53, c-Myc, heat shock protein 90 (HSP90) and tubulin [15, 17, 47–49, 51, 52]. In ovarian cancer, heightened expression of many HDAC class proteins has been described in 60–90 % of tumors analyzed and many histone and non-histone mediated alterations have been described that alter the balance in favor of cellular growth and survival [17, 53]. Our data confirm that LBH589 treatment, like SAHA, leads to significant acetylation of both histone and a non-histone protein. While therapy with SAHA led to decreases in Aurora-A expression, LBH589 failed to modify the expression levels. LBH589 treatment led to significant decreases in cell viability at lower concentrations than that observed with SAHA suggesting a higher potency. This activity in a spectrum of immortalized ovarian cancer cell lines confirms the experience of other investigators using other HDAC inhibitors [16, 17, 22]. Though some investigators have suggested Aurora-A may modulate HDAC inhibition of cancer cell proliferation [15], our data suggest LBH589 mediates anti-tumor effects via alternative mechanisms. Collectively, we observed that LBH589 exerts potent cancer cell control mediated through histone and non-histone molecular modifications.

While the exact mechanism HDAC inhibition employs to induce cell cycle arrest and apoptosis of ovarian cancer cells remains elusive, much preclinical data supports that HDAC inhibition synergizes with many cytotoxic chemotherapies including paclitaxel, carboplatin and docetaxel [25, 47, 54–57]. Investigators have hypothesized that synergy may be due to both histone hyperacetylation fostering intercalation of platinum as well as the heightened acetylated tubulin stabilization reinforced by both taxanes and HDAC inhibitors [17]. Others have suggested that HDAC inhibition potentiates cytotoxic chemotherapies by increasing double stranded breaks, precluded homologous repair and blocking the phosphotidylinositol 3-kinase (PI3K) pathway in in vitro ovarian cancer cells [57]. Recent studies have also implicated modulation of the multidrug resistance protein (MDR1), epidermal growth factor receptor (EGFR) and tumor initiating cells in order to facilitate complementary action with both targeted and cytotoxic therapeutics [25, 58, 59].

The article "Influence of a novel histone deacetylase inhibitor panobinostat (LBH589) on the growth of ovarian cancer" was published in 2016. Journal: J Ovarian Res.

These preclinical data provide context for our in vivo experiments utilizing a novel PDX model of serous ovarian cancer. Our studies confirmed that LBH589 precluded tumor growth compared to vehicle in three different tumors from women who underwent primary cytoreduction at our institution and suggest only a subset of high grade serous carcinomas will manifest heightened tumor regression if chemotherapy is administered in the setting of tonic HDAC inhibition. Importantly, we observed a tumorstatic response to P/C therapy in the OV3 PDXs only. In OV1 and OV2 PDXs P/C alone induced significant tumor regression. The observed toxicity of the treatments as manifested by mouse weight loss suggested that single agent LBH589 was well tolerated. These findings confirm numerous other studies that demonstrated that HDAC inhibitors were well tolerated by the animal models [17, 21, 22]. These observations provide rationale for the addition of HDAC inhibition in the setting of stable disease responses to conventional cytotoxic therapy. In the clinic, HDAC inhibition with SAHA (Vorinistat) has been combined with carboplatin and gemcitabine in a phase I trial that demonstrated partial responses in 6 out 7 women with recurrent ovarian cancer, though the trial was stopped early due to excessive toxicity [32].

## Conclusions

To our knowledge, this is the first report testing HDAC inhibition in concert with conventional chemotherapy in a PDX model derived from patients with high grade serous ovarian cancer. We believe this model has noteworthy clinical relevance and lends support to previous investigations utilizing immortalized cell lines. Our data showed that LBH589 had significant potency as an HDAC inhibitor, and that it induced hyperacetylation in histone and tubulin proteins while decreasing cell viability. The in vivo experiments confirmed a single agent tumorstatic effect of LBH589, and demonstrated, in a subset of our PDX models, an enhanced effect on tumor regression when combined with P/C. This investigation highlights HDAC inhibition with LBH589 as a promising avenue for innovating the treatment of ovarian cancer. Future study of LBH589 as a sequential or maintenance therapy will likely be of merit to further define how best to utilize this specialized therapeutic.

The article "Influence of a novel histone deacetylase inhibitor panobinostat (LBH589) on the growth of ovarian cancer" was published in 2016. Journal: J Ovarian Res.

## Abbreviations

DMEM: Dulbecco’s Modified Eagle’s Medium
HDAC: Histone deacetylase
HSP90: Heat shock protein 90
LBH589: Panobinostat
P/C: Paclitaxel and carboplatin
